The article "Effect of Xiaoyutang Combined with Intraperitoneal Heat Perfusion Chemotherapy on Immune Function, Circulating mir, Prognosis, and Survival of Postoperative Patients with Colorectal Cancer" was retracted in 2023. Reasons: signs of a paper mill; compromised peer review; unreliable results or conclusions.

# Effect of Xiaoyutang Combined with Intraperitoneal Heat Perfusion Chemotherapy on Immune Function, Circulating mir, Prognosis, and Survival of Postoperative Patients with Colorectal Cancer

**DOI:** 10.1155/2021/1619809

**Published:** 2021-12-14

**Authors:** Lingxia Li, Yunjiu Wang, Xiaowan Huang, Jian Sun, Jue Zhang

**Affiliations:** Shuguang Hospital Affiliated to Shanghai University of Traditional Chinese Medicine, China

## Abstract

**Objective:**

To explore the effects of Xiaoyutang combined with intraperitoneal heat perfusion chemotherapy on immune function, circulating Mir, and prognosis and survival of postoperative patients with colorectal cancer.

**Methods:**

A total of 96 patients with colorectal cancer who were treated in our hospital from May 2018 to August 2019 and followed up to August 2021 were selected as the study subjects. The patients were randomly divided into a control group and study group by a 1 : 1 random number table method, 48 cases in each group. Patients in the control group were given intraperitoneal thermal perfusion chemotherapy after surgery, and patients in the research group were treated with Xiaoyutang on this basis. The treatment cycle was 21 days, and all patients were treated for 3 consecutive cycles. The therapeutic efficacy, immune function (CD3^+^, CD4^+^, and CD4^+^/CD8^+^), circulating mir (mir-29a, mir-145, and mir-92a), prognosis, and survival of the two groups were compared.

**Results:**

After 3 cycles of treatment, ORR and DCR in the study group were higher than those in the control group (60.42% vs. 37.50%) and 85.42% vs. 66.67%, respectively, with statistical significance (*P* < 0.05). There were statistically significant differences in CD3^+^, CD4^+^, CD4^+^/CD8^+^, mir-29a, mir-145, and mir-92a time points and intergroup and intergroup interactions between the two groups (*P* < 0.05); the levels of CD3^+^, CD4^+^, and CD4^+^/CD8^+^ in the study group were higher than those in the control group after 1, 2, and 3 cycles of treatment (*P* < 0.05); the expressions of mir-29a, mir-145, and mir-92a were significantly lower than those in the control group (*P* < 0.05). By the end of follow-up, 3 cases were lost to follow-up in the study group and 5 cases in the control group. The recurrence rate and mortality of the study group were lower than those of the control group at 1- and 2-year follow-up (*P* > 0.05), and the mean survival time of patients in the study group was higher than that in the control group; the differences were statistically significant (*χ*^2^ = 5.151, *P* = 0.023).

**Conclusion:**

Xiaoyutang combined with peritoneal heat perfusion chemotherapy has a good postoperative effect on patients with colorectal cancer, which can effectively improve the immune function and circulating Mir of patients with colorectal cancer, reduce tumor recurrence, and improve the prognosis of patients.

The article "Effect of Xiaoyutang Combined with Intraperitoneal Heat Perfusion Chemotherapy on Immune Function, Circulating mir, Prognosis, and Survival of Postoperative Patients with Colorectal Cancer" was retracted in 2023. Reasons: signs of a paper mill; compromised peer review; unreliable results or conclusions.

## 1. Introduction

The causes of colorectal cancer are mostly related to lifestyle, genetics, colorectal adenoma, and other factors. Its early symptoms are not obvious. With the progress of the disease, there is no opportunity for surgical treatment in the late stage. The survival rate within 5 years is only about 5%, which can seriously threaten the life and health of patients [1]. Surgical treatment is one of the treatment methods for patients with colorectal cancer, but surgery cannot eradicate tumor cells, resulting in residual tumor metastasis and recurrence, which affects the prognosis. Chemotherapy is an effective adjuvant treatment for colorectal cancer after operation, but affected by the peritoneal plasma barrier, only a small number of chemotherapy drugs can enter the abdominal cavity through intravenous chemotherapy, so the killing effect of free cancer cells in the abdominal cavity is poor [2]. Intraperitoneal thermal perfusion is an efficient chemotherapy regimen for gastrointestinal tumors, which can effectively control the recurrence and metastasis of cancer cells in the abdominal cavity [3]. Although the antitumor effect of intraperitoneal hyperthermic perfusion chemotherapy is strong, the toxic effect of chemotherapy can cause immune dysfunction. Traditional Chinese medicine can regulate the postoperative immune abnormalities of colorectal cancer through dialectical treatment, improve the body's immunity, and improve the prognosis of tumor patients [4]. At present, there are few reports on the impact of integrated traditional Chinese and Western medicine on the immune function of patients with colorectal cancer. Based on this, this study investigated the effects of Xiaoliu Decoction combined with intraperitoneal thermal perfusion chemotherapy on immune function, circulating Mir, and prognostic survival of postoperative patients with colorectal cancer, in order to provide reference for the treatment of rectal cancer. The results are as follows.

## 2. Information and Methods

### 2.1. General Information

96 patients with colorectal cancer treated in our hospital from May 2018 to August 2019 and followed up to August 2021 were selected as the research objects. The case inclusion criteria are as follows: (1) meet the standard of China colorectal cancer diagnosis and treatment code (2017 version) [5]; (2) no liver metastasis or distant metastasis was found by CT or B-ultrasound; (3) estimated survival time > 6 months; and (4) the clinical data are complete. The exclusion criteria are as follows: (1) patients with important organ diseases; (2) other malignant tumors; (3) severe infectious diseases; (4) persons with cognitive impairment; and (5) unable to cooperate with the researcher. The selected patients were randomly divided into a control group and study group at 1 : 1. There was no significant difference in baseline data between the two groups (*P* > 0.05) (Table 1). This study was approved by the medical ethics committee of the college.

The article "Effect of Xiaoyutang Combined with Intraperitoneal Heat Perfusion Chemotherapy on Immune Function, Circulating mir, Prognosis, and Survival of Postoperative Patients with Colorectal Cancer" was retracted in 2023. Reasons: signs of a paper mill; compromised peer review; unreliable results or conclusions.

### 2.2. Method

The patients in the control group were treated with intraperitoneal thermal perfusion after operation. After the cancer focus was removed during the operation, a silicone tube was placed in the pelvic cavity and upper abdominal wall, respectively, connected to the thermal perfusion chemotherapy instrument, and the incision was sutured. The chemotherapy drug is composed of 1000 mg 5-fluorouracil+80 mg cisplatin+1500 ml 0.9% sodium chloride injection. The flow rate of perfusion chemotherapy is 150 ml/min, and the temperature in the abdominal cavity is maintained at 43 ± 0.5°C. After operation, a special drainage device was used to remove the coagulation block, fibrous tissue, and exfoliated necrotic tissue in the drainage tube. At the same time, on the first day after operation, thermoperfusion chemotherapy was carried out again for 30 minutes, once a week, 3 weeks as a cycle, and 3 consecutive cycles of treatment.

The study group was treated with Xiaoliu Decoction on the basis of the former. Xiaoliu Decoction consists of 15 g Astragalus membranaceus, 15 g Codonopsis pilosula, 15 g arrowhead mushroom, 15 g Scutellaria barbata, 20 g coix seed, 12 g fufangteng, 6 g Tianqi, and 6 g Ziheche. The above Chinese medicinal materials are decocted to 300 ml with water, one dose a day, and take warmly are taken twice in the morning and evening. Continuous treatment was done for 3 cycles.

### 2.3. Observation Indicators

1. Efficacy: the efficacy was evaluated according to the evaluation criteria of complete remission (CR), partial remission (PR), disease stability (SD), and disease progression (PD) in RECIST 1.1 solid tumor efficacy evaluation criteria [6]. Objective response rate (ORR) = (Cr + PR)/*n* × 100%; disease control rate (DCR) = (Cr + PR + SD)/*n* × 100%
2. Immune function: 2 ml peripheral venous blood was taken before treatment, 1 cycle, 2 cycle, and 3 cycle, respectively, and the levels of CD3^+^, CD4^+^, and CD4^+^/CD8^+^ were detected by flow cytometry (Beckman, USA)
3. Circulating Mir: 2 ml of peripheral venous blood was extracted before treatment, cycle 1, cycle 2, and cycle 3, respectively, and the expressions of mir-29a, mir-145, and mir-92a were detected by real-time fluorescence quantitative method
4. Prognosis: after treatment, the patients were followed up for two years by telephone and outpatient and family visits. The deadline for follow-up was August 31, 2021

The article "Effect of Xiaoyutang Combined with Intraperitoneal Heat Perfusion Chemotherapy on Immune Function, Circulating mir, Prognosis, and Survival of Postoperative Patients with Colorectal Cancer" was retracted in 2023. Reasons: signs of a paper mill; compromised peer review; unreliable results or conclusions.

### 2.4. Statistical Analysis

The statistical software SPSS22.0 was used to process the data, and the counting data (*n*, %) represented independent samples *χ*^2^ test and rank sum test. The measurement data conforming to the normal distribution are represented by ($\bar{x}\pm s$), and independent sample *t*-test is performed. The immune function and circulating Mir indexes at different times were analyzed by repeated measurement analysis of variance. The prognosis was analyzed by the Kaplan Meier survival curve, and the difference was tested by log rank (Mantel-Cox). *P* < 0.05 was statistically significant.

## 3. Results

### 3.1. Comparison of Short-Term Efficacy between the Two Groups

After 3 cycles of treatment, the ORR in the study group was higher than that in the control group (60.42% vs. 37.50%), and the DCR was higher than that in the control group (85.42% vs. 66.67%) (*P* < 0.05) (see Table 2).

### 3.2. Comparison of Immune Function between the Two Groups

There were significant differences in the time point of CD3^+^, CD4^+^, and CD4^+^/CD8^+^ and the interaction between the two groups (*P* < 0.05). After 1, 2, and 3 cycles of treatment, the levels of CD3^+^, CD4^+^, and CD4^+^/CD8^+^ in the study group were higher than those in the control group (*P* < 0.05) (see Table 3).

### 3.3. Comparison of Circulating Mir Indexes between the Two Groups

The time point of mir-29a, mir-145, and mir-92a; the time point between groups; and the interaction between groups were statistically significant (*P* < 0.05). After 1, 2, and 3 cycles of treatment, the expressions of mir-29a, mir-145, and mir-92a in the study group were significantly lower than those in the control group (*P* < 0.05) (see Table 4).

### 3.4. Analysis and Comparison of Prognosis and Survival

At the end of follow-up, 3 cases in the study group and 5 cases in the control group were lost. The recurrence rate and mortality in the study group were lower than those in the control group (*P* > 0.05), and the average survival time of patients in the study group was higher than that in the control group. Log rank test showed that the differences were statistically significant (*χ*^2^ = 5.151, *P* = 0.023) (see Tables 5 and 6 and Figure 1).

## 4. Discussion

Surgical resection is effective in the treatment of colorectal cancer, but surgery cannot completely remove the tumor cells, and the residual tumor cells can enter the blood circulation through metastasis and dissociation, resulting in cell residue and tumor recurrence, which affects the prognosis of patients. Postoperative adjuvant chemotherapy can effectively kill micrometastasis, control tumor metastasis and recurrence, and then prolong the survival time of patients. However, there are still disputes about the mode of chemotherapy [7]. Intraperitoneal hyperthermic perfusion chemotherapy is a highly selective local chemotherapy scheme, which perfuses heated chemotherapy drugs into the abdominal cavity through systemic circulation and washes and kills tumor cells free in the abdominal cavity through the hyperthermic effect and tumor inactivation of chemotherapy solution, so as to reduce the recurrence and metastasis of tumor after operation [8]. Moreover, intraperitoneal hyperthermic perfusion chemotherapy can make the tumor vascular endothelial cells closely connected, reduce the gap between blood vessels, and thicken the vascular wall, so as to control tumor metastasis and the growth of new blood vessels and enhance the antitumor effect [9]. Although the antitumor effect of intraperitoneal hyperthermic perfusion chemotherapy is strong, the toxic effect of chemotherapy can cause immune dysfunction.

The article "Effect of Xiaoyutang Combined with Intraperitoneal Heat Perfusion Chemotherapy on Immune Function, Circulating mir, Prognosis, and Survival of Postoperative Patients with Colorectal Cancer" was retracted in 2023. Reasons: signs of a paper mill; compromised peer review; unreliable results or conclusions.

Traditional Chinese medicine can start from the whole and regulate the dysfunction of Zang Fu organs by syndrome differentiation, so as to achieve the role of strengthening the foundation, eliminating swelling and dispersing knots. According to traditional Chinese medicine, colorectal cancer belongs to the category of “intestine Qin” and “blood in stool.” It is the main cause of deficiency of qi and blood, deficiency of the spleen and stomach, phlegm, qi, and blood stasis [10]. It is recorded in the medical records of external evidence that “deficiency of healthy qi leads to diagenesis”; “Jing Yue Quan Shu” said: “eating incoherent, resulting in damage to the spleen and stomach.” If the viscera are weak and the spleen fails to function properly, the phlegm is blocked, the biochemical source is lacking, and it accumulates in the intestine, which is called intestinal Qin. At the same time, the six exogenous factors of the body lead to the weakness of healthy qi, the invasion of evil qi, the accumulation of phlegm and poison, and the injury of emotion, resulting in the stagnation of liver qi and poor blood circulation, which will lead to tumors [11]. Therefore, the key points for the treatment of this disease are strengthening the body, eliminating swelling and evil, promoting blood circulation, and removing blood stasis. Xiaoliu Decoction is composed of Astragalus membranaceus, Codonopsis pilosula, Pleurotus ostreatus, Scutellaria barbata, coix seed, fufangteng, Tianqi, and Ziheche. Astragalus membranaceus, Codonopsis pilosula, and Ziheche are all king drugs; Pleurotus ostreatus, Scutellaria barbata, fufangteng, and Tianqi are minister drugs; and coix seed is an auxiliary drug. Pharmacology of traditional Chinese medicine has proved that Astragalus membranaceus, Codonopsis pilosula, and Ziheche are important drugs for supplementing qi, which have the effects of promoting blood circulation, supplementing qi, eliminating evil, and strengthening health. Arrowhead mushroom can eliminate carbuncle and disperse knot; Scutellaria barbata can clear away heat and toxin, promote blood circulation, remove blood stasis, reduce swelling, relieve pain, and fight cancer; Fufangteng has the effect of hemostasis and stasis elimination. In addition, Tianqi can dissipate blood stasis and detumescence, and the combination of the four can promote blood circulation, remove blood stasis, and dispel evil and detumescence [12]. Coix seed has the effects of strengthening the spleen, stopping diarrhea, detoxifying, and dispersing knot. It is mainly used for diarrhea due to spleen deficiency, intestinal carbuncle, cancer, and so on. Therefore, the whole prescription can be used to replenish qi and blood, support righteousness, dispel evil, eliminate swelling and knot, strengthen the spleen, and diuresis. Modern pharmacological studies have confirmed that Astragalus membranaceus has anticancer effect, killing cell activity, improving body immunity, and improving the quality of life of tumor patients. Codonopsis pilosula contains a variety of trace alkaloids, which can effectively increase the tumor volume and improve the body's immunity. In this study, after treatment, the ORR and DCR of the study group were higher than those of the control group, the recurrence rate and mortality were lower than those of the control group, and the survival time of the study group was higher than that of the control group. The results suggest that the antitumor effect of Xiaoliu Decoction combined with intraperitoneal thermal perfusion chemotherapy is better than that of intraperitoneal thermal perfusion chemotherapy alone.

The article "Effect of Xiaoyutang Combined with Intraperitoneal Heat Perfusion Chemotherapy on Immune Function, Circulating mir, Prognosis, and Survival of Postoperative Patients with Colorectal Cancer" was retracted in 2023. Reasons: signs of a paper mill; compromised peer review; unreliable results or conclusions.

Cellular immunity is an important part of the immune system, and the abnormal immune system caused by surgical trauma can have a serious impact on the prognosis of tumor patients. Studies have confirmed that patients' immune function can affect tumor recurrence to a certain extent [13]. T lymphocytes are the main component of cellular immunity, and their number and proportion can directly reflect the state of immune function. CD3^+^ mainly exists on the cell surface and can participate in T cell activation signal transduction and initiate immune response. CD4^+^ can assist the expression of T cells and further improve the antitoxic ability of the body. In addition, CD4^+^/CD8^+^ can reflect the dynamic balance of the body, and the greater the CD4^+^/CD8^+^ ratio, the stronger the antiobstruction ability of immune cells. In this study, the levels of CD3^+^, CD4^+^ and CD4^+^/CD8^+^ in the study group were higher than those in the control group after 1, 2, and 3 cycles of treatment. The results are consistent with the conclusions of Jingchun [14], suggesting that Xiaoliu Decoction combined with intraperitoneal thermal perfusion chemotherapy can effectively improve the postoperative immune function of patients with colorectal cancer. The reasons are as follows: during intraperitoneal thermal perfusion chemotherapy, the increase of chemotherapy fluid temperature can promote the increase of tumor cell antigenicity, activate the immune function, and promote the immune response. Moreover, hyperthermic perfusion chemotherapy can increase the ability of intravascular natural killer cells in cancer tissues and improve immune function to a certain extent [15].

In addition, mirna is a noncoding small RNA, which can regulate gene expression and participate in the occurrence and development of tumor diseases. And it has been confirmed by research. Mirna has an effect on tumor proliferation, invasion, metastasis, and differentiation [16]. It has the functions of oncogene and tumor suppressor gene. When the target gene of mirna is oncogene, it can inhibit body lesions under normal conditions, but when the expression of mirna is lower than the normal level, the inhibitory effect of oncogene can be weakened, resulting in tumor metastasis and recurrence. When the target of mirna is tumor suppressor gene, its increased expression can hinder the expression of oncogene and promote the occurrence and metastasis of tumor. Mir-29a, mir-145, and mir-92a belong to mirna type. In this study, the expression of mir-29a, mir-145, and mir-92a in the study group was significantly lower than that in the control group after 1, 2, and 3 cycles of treatment. It is suggested that Xiaoliu Decoction combined with intraperitoneal thermal perfusion chemotherapy can improve circulating Mir in patients with colorectal cancer.

In conclusion, Xiaoliu Decoction combined with intraperitoneal thermal perfusion chemotherapy has a good curative effect on patients with colorectal cancer. It can effectively improve the immune function and circulating Mir of patients with colorectal cancer, reduce tumor recurrence, and improve the prognosis of patients. The deficiency of this study is that there are few research samples and the follow-up time of patients is relatively short, so it still needs to be further verified by large-scale research.

The article "Effect of Xiaoyutang Combined with Intraperitoneal Heat Perfusion Chemotherapy on Immune Function, Circulating mir, Prognosis, and Survival of Postoperative Patients with Colorectal Cancer" was retracted in 2023. Reasons: signs of a paper mill; compromised peer review; unreliable results or conclusions.

## Figures and Tables

**Figure 1:** Comparison of survival time between the two groups.

**(a):** 

Group	Gender		Age (years)	BMI (kg/m^2^)	Tumor location		TNM staging	
	Male	Female			Colon	Rectum	Phase III	Phase IV
Research group (48)	26	22	51.24 ± 5.62	23.56 ± 3.52	25 (52.08)	23 (47.92)	35 (72.92)	13 (27.08)
Control group (48)	28	20	52.48 ± 5.10	23.82 ± 3.22	28 (58.33)	20 (41.67)	37 (77.08)	11 (22.92)
*T*/*χ*^2^ value	0.169		1.132	0.378	0.379		0.222	
*P* value	0.681		0.261	0.707	0.538		0.637	

**(b):** 

Degree of differentiation			Complication			
Low differentiation	Medium differentiation	High differentiation	Diabetes	Heart disease	Hypertension	Respiratory diseases
15 (31.25)	26 (54.17)	7 (14.58)	8 (16.67)	5 (10.42)	12 (25)	6 (12.5)
17 (35.42)	23 (47.92)	8 (16.67)	10 (20.83)	7 (14.58)	10 (20.83)	8 (16.67)
-0.198			-0.200			
0.843			0.841			

**Table 2:** Comparison of short-term curative effects between the two groups.

Group	Cases	CR	PR	SD	PD	ORR	DCR
Research group	48	5 (10.42)	24 (50.00)	12 (25.00)	7 (14.58)	29 (60.42)	41 (85.42)
Control group	48	1 (2.08)	17 (35.42)	14 (29.17)	16 (33.33)	18 (37.50)	32 (66.67)
*Z*/*χ*^2^值	—	-2.655				5.044	4.631
*P* value		0.008				0.025	0.031

**Table 3:** Comparison of immune function between the two groups.

Index	Group	Before treatment	Treatment 1 cycle	Treatment 2 cycle	Treatment 3 cycle	*F* value	*P* value
CD3^+^ (%)	Research group (48)	56.84 ± 5.20	58.37 ± 5.23	60.70 ± 5.49	64.24 ± 5.62	*F*_*Time* *point*_ = 98.538 *F*_*Interactive*_ = 24.983 *F*_*Between* *groups*_ = 12.778	*P*_*Time* *point*_ < 0.001 *P*_*Interactive*_ = 0.004 *P*_*Between* *group*_ = 0.001
	Control group (48)	55.97 ± 5.72	55.86 ± 5.10	56.79 ± 5.34	58.36 ± 5.49		
	*T* value	0.780	2.381	3.537	5.185		
	*P* value	0.438	0.019	0.001	<0.001		

CD4^+^ (%)	Research group (48)	31.52 ± 3.56	35.82 ± 3.76	38.74 ± 4.53	44.83 ± 5.10	*F*_*Time* *point*_ = 642.209 *F*_*Interactive*_ = 64.141 *F*_*Between* *groups*_ = 33.010	*P*_*Time* *point*_ < 0.001 *P*_*Interactive*_ < 0.001 *P*_*Between* *group*_ < 0.001
	Control group (48)	30.95 ± 3.01	32.35 ± 3.11	34.55 ± 4.10	37.64 ± 4.34		
	*T* value	0.847	4.927	4.751	7.439		
	*P* value	0.399	<0.001	<0.001	<0.001		

CD4^+^/CD8^+^	Research group (48)	1.16 ± 0.09	1.35 ± 0.22	1.54 ± 0.32	1.62 ± 0.37	*F*_*Time* *point*_ = 165.242 *F*_*Interactive*_ = 12.158 *F*_*Between* *groups*_ = 15.967	*P*_*Time* *point*_ < 0.001 *P*_*Interactive*_ = 0.001 *P*_*Between* *group*_ < 0.001
	Control group (48)	1.15 ± 0.11	1.18 ± 0.19	1.30 ± 0.25	1.41 ± 0.28		
	*T* value	0.487	4.052	4.095	3.136		
	*P* value	0.627	<0.001	<0.001	0.002		

The article "Effect of Xiaoyutang Combined with Intraperitoneal Heat Perfusion Chemotherapy on Immune Function, Circulating mir, Prognosis, and Survival of Postoperative Patients with Colorectal Cancer" was retracted in 2023. Reasons: signs of a paper mill; compromised peer review; unreliable results or conclusions.

**Table 4:** Comparison of circulating Mir indexes between the two groups.

Index	Group	Before treatment	Treatment 1 cycle	Treatment 2 cycle	Treatment 3 cycle	*F* value	*P* value
Mir-29a	Research group (48)	0.44 ± 0.13	0.15 ± 0.06	0.13 ± 0.02	0.11 ± 0.04	*F*_*Time* *point*_ = 513.006 *F*_*Interactive*_ = 29.368 *F*_*Between* *groups*_ = 103.863	*P*_*Time* *point*_ < 0.001 *P*_*Interactive*_ < 0.001 *P*_*Between* *group*_ < 0.001
	Control group (48)	0.41 ± 0.07	0.37 ± 0.05	0.32 ± 0.09	0.22 ± 0.12		
	*T* value	1.408	19.515	14.278	6.025		
	*P* value	0.163	<0.001	<0.001	<0.001		

Mir-145	Research group (48)	0.55 ± 0.07	0.24 ± 0.08	0.20 ± 0.10	0.10 ± 0.05	*F*_*Time* *point*_ = 1276.227 *F*_*Interactive*_ = 123.693 *F*_*Between* *groups*_ = 154.599	*P*_*Time* *point*_ < 0.001 *P*_*Interactive*_ < 0.001 *P*_*Between* *group*_ < 0.001
	Control group (48)	0.58 ± 0.14	0.43 ± 0.06	0.42 ± 0.13	0.34 ± 0.06		
	*t* value	1.328	13.164	9.293	21.290		
	*P* value	0.187	<0.001	<0.001	<0.001		

Mir-92a	Research group (48)	0.58 ± 0.12	0.40 ± 0.12	0.36 ± 0.11	0.27 ± 0.02	*F*_ 时 点 _ = 456.037 *F*_*Interactive*_ = 11.921 *F*_*Between* *groups*_ = 16.916	*P*_*Time* *point*_ < 0.001 *P*_*Interactive*_ = 0.001 *P*_*Between* *group*_ < 0.001
	Control group (48)	0.55 ± 0.12	0.52 ± 0.10	0.42 ± 0.05	0.35 ± 0.10		
	*t* value	1.225	5.322	3.440	5.435		
	*P* value	0.224	<0.001	0.001	<0.001		

**Table 5:** Comparison of survival between the two groups.

Grouping	Number of cases	Recurrence (cases)		Death (cases)	
		1-year recurrence	2-year recurrence	1-year death	2-year death
Research group	45	9 (20.00)	20 (44.44)	8 (17.78)	16 (35.56)
Control group	43	15 (34.88)	27 (62.79)	12 (27.91)	24 (55.81)
*Χ* ^2^ value	—	2.456	2.974	1.285	3.64
*P* value		0.117	0.085	0.257	0.056

**Table 6:** Mean and median survival time.

Grouping	Average value (*E*)				Log rank	
	Estimate	Standard error	95% confidence interval			
			Lower limit	Upper limit	*Χ* ^2^	*P*
Research group	18.908	1.038	16.873	20.942	5.151	0.023
Control group	16.766	1.520	13.786	19.746		
Totality	19.123	1.039	17.087	21.159		

## Data Availability

The data used to support this study are available from the corresponding author upon request.
